The article "Classification for Memory Activities: Experiments and EEG Analysis Based on Networks Constructed via Phase-Locking Value" was published in 2022. Journal: Comput Math Methods Med.

# Classification for Memory Activities: Experiments and EEG Analysis Based on Networks Constructed via Phase-Locking Value

**DOI:** 10.1155/2022/3878771

**Published:** 2022-06-28

**Authors:** Jing Xi, Xiao-Lin Huang, Xing-Yan Dang, Bin-Bin Ge, Ying Chen, Yun Ge

**Affiliations:** ^1^School of Electronic Science and Engineering, Nanjing University, Nanjing 210023, China; ^2^The Affiliated Tumor Hospital of Nantong University, Nantong 226361, China

## Abstract

Electroencephalogram (EEG) plays a crucial role in the study of working memory, which involves the complex coordination of brain regions. In this research, we designed and conducted series of experiments of memory with various memory loads or target forms and collected behavioral data as well as 32-lead EEG simultaneously. Combined with behavioral data analysis, we segmented EEG into slices; then, we calculated phase-locking value (PLV) of Gamma rhythms between every two leads, conducted binarization, constructed brain function network, and extracted three network characteristics of node degree, local clustering coefficient, and betweenness centrality. Finally, we inputted these network characteristics of all leads into support vector machines (SVM) for classification and obtained decent performances; i.e., all classification accuracies are greater than 0.78 on an independent test set. Particularly, PLV application was restricted to the narrow-band signals, and rare successful application to EEG Gamma rhythm, defined as wide as 30-100 Hz, had been reported. In order to address this limitation, we adopted simulation on band-pass filtered noise with the same frequency band as Gamma to help determine the PLV binarizing threshold. It turns out that network characteristics based on binarized PLV have the ability to distinguish the presence or absence of memory, as well as the intensity of the mental workload at the moment of memory. This work sheds a light upon phase-locking investigation between relatively wide-band signals, as well as memory research via EEG.

## 1. Introduction

Working memory (WM) [1] is a memory system that stores and processes information for a short time. It plays a key role in many complex cognitive tasks such as language comprehension, learning, and reasoning.

In addition to traditional psychoanalysis and behavioral data analysis, the use of functional magnetic resonance imaging (fMRI), electroencephalography, and other quantifiable techniques for working memory research has gradually become the mainstream. Among them, electroencephalography is more and more popular because it can capture dynamics in memorizing activity time frame, which spans hundreds of milliseconds to a few seconds, and it directly measures neural electrical activities. Moreover, EEG provides critical information from four dimensions, i.e., space, time, power, and phase [2, 3].

The article "Classification for Memory Activities: Experiments and EEG Analysis Based on Networks Constructed via Phase-Locking Value" was published in 2022. Journal: Comput Math Methods Med.

Conventionally, EEG analysis includes time-domain analysis, frequency-domain analysis, and time-frequency-domain analysis. Time-domain methods extract features directly from raw signals of EEG or a decomposed signal such as empirical mode decomposition (EMD). Well-known time-domain features (TDFs) include mean, variance, mode, median, and kurtosis. For example, Koivisto et al. conducted an ERP analysis on the EEG data and found that frontal regions contributed to higher-level cognitive processes by calculating the peak amplitude of the average waveform [4]. Frequency-domain analysis focuses on characteristics extracted from power spectrum of EEG. Perlis et al. studied the power spectrum of the EEG of insomnia patients and confirmed that Beta/Gamma activity was increased in primary insomnia [5]. In research of young men's working memory, Guevara et al. reported that the EEG power of the delta band was higher than the power of the Gamma band, and the right frontal area was more involved in the processing of working memory [6]. Meltzer et al. found that the memory loading effect of power spectral energy showed different characteristics in different brain regions; for example, Theta and Alpha wave energy increased mainly in the front central region with a positive loading effect and decreased in the occipital, dorsal frontal, and parietal lobes with a negative loading effect [7]. Time-frequency analysis combines time-domain with frequency-domain analysis by sliding or scaling a time window. Schneider et al. used time-frequency analysis named as event-related spectral perturbation to analyze EEG in working memory stage and found that separate excitatory and inhibitory processes underlay the deployment of attention on the level of working memory representations [8].

In recent years, brain connectivity and brain network analyses, which focus on coordinated functions of different brain regions, have become more and more popular. As for EEG, indices that measure relationship between signals collected from different positions or leads are firstly extracted, and then, connectivity or network attributes are further investigated. The relationship measures vary from time-domain linear correlation coefficient, frequency-domain coherence, to nonlinear-domain phase synchronization parameters. For example, Joudaki et al. experimented on 32 subjects, extracted functional networks of three different sizes, and found that the network size should be considered in any comparison of networks across studies [9]. Donner and Nieuwenhuis have reported that postsynaptic potentials and network connections evolved dynamically with positive feedback over time during attention and learning, resulting in “the rich getting richer” [10, 11].

The article "Classification for Memory Activities: Experiments and EEG Analysis Based on Networks Constructed via Phase-Locking Value" was published in 2022. Journal: Comput Math Methods Med.

The parameters in the time domain, frequency domain, or time-frequency domain are all linear parameters and are easily affected by signal amplitude, and the amplitude of EEG is easily overwhelmed by interference due to its low signal-to-noise ratios [2]. Whereas phase contains the nonlinear information of the signal and is independent of the amplitude, therefore, it can provide an important supplement [2]. Previous studies have shown that there is a widespread phase-locking phenomenon in neural activities, and phase-locking value (PLV), which measures phase locking, has been successfully applied to LFP and spikes. For example, based on the PLV difference between events, Gonuguntla and Kim presented a framework to find significant functional network (SFN) corresponding to its event, then applied it to the DEAP dataset, and obtained the SFNs associated with emotions [12]. In this study, we adopted PLV to measure the phase synchronization between two EEG series from different leads.

Support vector machine (SVM) [13] is a machine learning model with nonlinear classification ability and has been successfully applied to EEG classification in various scenes. For example, Turnip et al. used SVM separate lying subjects from the innocent one based on signal P300 [14, 15]. In this work, we tried SVM for classification.

In this work, we designed and conducted series of experiments concerning memory and collected behavioral data as well as 32-lead EEG simultaneously. Combined with behavioral data analysis, we segmented EEG to slices; then, we calculated Gamma rhythm PLV between every two leads, conducted binarization, constructed brain function network, and extracted three network characteristics of node degree, local clustering coefficient, and betweenness centrality. Finally, we inputted these network characteristics of all leads into SVMs for classification and obtained descent performances. Specifically, considering that PLV was restricted to single-frequency or narrow-band signal analysis [16, 17] and rare successful application to EEG Gamma rhythm had been reported, we adopted simulation on band-pass filtered noise with the same frequency band as Gamma to help determine the PLV binarizing threshold. It turns out that network characteristics based on binarized PLV have the ability to distinguish the presence or absence of memory, as well as the intensity of the mental workload at the moment of memory.

## 2. Method

### 2.1. The Phase-Locking Value

Given two simultaneously collected signals of length *N*, *x*_1_(*t*_*l*_), and *x*_2_(*t*_*l*_) (*l* = 1, 2, ⋯, *N*), corresponding instantaneous phase series *φ*_1_(*t*_*l*_) and *φ*_2_(*t*_*l*_) are first calculated via Hilbert transformation [18]. Then, PLV which was originally proposed by Lachaux et al. between *x*_1_ and *x*_2_ is defined as [19]

(1) $$\begin{array}{c} {\text{PLV}}_{12}=\frac{1}{N}\left|\overset{N}{\underset{l=1}{\sum }}\exp\left(j\left(\Delta \varphi_{12}\left(t_{l}\right)\right)\right)\right|, \end{array}$$

where Δ*φ*_12_(*t*_*l*_) = *φ*_1_(*t*_*l*_) − *φ*_2_(*t*_*l*_) represents the instantaneous phase difference between *x*_1_ and *x*_2_ and *j* represents imaginary unit. PLV ranges between 0 and 1, in which 0 indicates Δ*φ*  randomly distributed on a unity circle, i.e., non-phase locking, and 1 indicates Δ*φ* keeping constant, i.e., perfect phase locking. However, PLV works well only for single-frequency or narrow-band signals [17]. For signals with a wide frequency band, the ability of PLV to detect phase lock greatly deteriorates; that is, a higher PLV is not available even when there does exist phase locking [19]. As a result, the threshold to determine whether there is a phase locking or not, i.e., a binary judgment, is difficult to define. In this manuscript, by generating simulating series using filtered noises, which are consistent with EEG in frequency, we analyzed the distributions of simulating series' PLVs for different cases and then determined the binarization threshold based on them. In following experimental data analysis, we would focus on the binary PLV, denoted as *a*_*ij*_, in which *i*, *j* represent different EEG lead labels and the values 0 and 1 indicate non-phase locking and phase locking, respectively.

The article "Classification for Memory Activities: Experiments and EEG Analysis Based on Networks Constructed via Phase-Locking Value" was published in 2022. Journal: Comput Math Methods Med.

### 2.2. Brain Network Characteristics

After the binary PLVs were obtained between every two EEG leads, we constructed the network, treating each scalp electrode as a node and each nonzero *a*_*ij*_ as a link (or edge) between lead *i* and lead *j*.

We mainly investigated three network characteristics: node degree, clustering coefficient, and betweenness centrality [2, 9].

The degree of the *i*th node, denoted as *D*_*i*_, is defined as [20]

(2) $$\begin{array}{c} D_{i}=\underset{j\in G}{\sum }a_{ij}. \end{array}$$

As defined, *D*_*i*_ represents the total number of edges connecting the *i*th node with others in graph *G*, which embraces all leads and thus measures the connectivity of the node *i* and partly reflects the importance of the node in the network.

*C*_*i*_, the local clustering coefficient of node *i*, is defined as [21–23]

(3) $$\begin{array}{c} C_{i}=\frac{E_{i}}{k_{i}\left(k_{i}-1\right)/2}, \end{array}$$

in which *E*_*i*_ represents the number of edges among the neighbors of node *i* and *k*_*i*_ is the number of neighbors of node *i*. Herein, neighbors of node *i* refer to those nodes connecting directly with node *i*, regardless of the spatial distance. In fact, *E*_*i*_ gets to the minimum of 0, when there is no connection among the neighbors, and reaches the maximum of (*k*_*i*_(*k*_*i*_ − 1))/2, when all neighbors are connected with each other, i.e., full-connected. Therefore, clustering coefficient *C*_*i*_ depicts the actual edge ratio to potentially most edges in the neighborhood, thus reflecting local connectivity. *C*_*i*_ ranges between 0 and 1.

Betweenness centrality is an indicator of the centrality size of nodes in the graph. In an undirected binary network, the betweenness centrality of the *i*th node is defined as [24, 25]

(4) $$\begin{array}{c} b_{i}=\underset{m,n\in G,m\neq n\neq i}{\sum }\frac{\sigma_{mn}\left(i\right)}{\sigma_{mn}}, \end{array}$$

where *σ*_*mn*_ is the number of shortest paths between node *m* and node *n* and *σ*_*mn*_(*i*) is the number of shortest paths between node *m* and *n* that pass through node *i*. Betweenness centrality also ranges from 0 to 1. The more times a node acts as an “intermediary,” the greater its betweenness centrality, which means that more information flows to the node.

### 2.3. Classification

Various previous researches have demonstrated the validity of SVM application to EEG [15, 25, 26]. Therefore, we adopted SVM to realize classifications in this manuscript.

After obtaining aforementioned three network characteristics for 32 electrodes, we input the 96-dimention vector into a SVM with a RBF kernel for classification. Two crucial hyperparameters, namely, the penalty factor *C* and the kernel function parameter *γ*, were optimized by grid searching. Model outputting is the classified label, the number of which depends on the specific task, which will be described in Section 5.2.

### 2.4. The Overall Flow Chart

The overall flow chart of our method is shown in Figure 1.

## 3. Simulation

As aforementioned, for signals with wide frequency band, it is difficult to obtain a low PLV even when there does exit phase locking [17, 27]. In this manuscript, simulation was used to resolve the problem, namely, to obtain the threshold for PLV binarization. Without loss of generality, all simulating series in this manuscript, denoted as *s*(*t*), were generated by band-pass filtering normalized Gaussian white noise *σ*(*t*), which has zero-mean and one-standard deviation. In order to keep consistent with the subsequent experimental EEG analysis, the sampling rate in simulation is set to 1 KHz, and the series length used to calculate the PLV is 1 s. Besides, the selected frequency band depends on the EEG rhythm in following analysis. In this work, Gamma rhythm was concerned; therefore, 30 Hz-100 Hz band-pass filtering was adopted.

The article "Classification for Memory Activities: Experiments and EEG Analysis Based on Networks Constructed via Phase-Locking Value" was published in 2022. Journal: Comput Math Methods Med.

Actually, there are alternative methods like constructing surrogates by shuffling time series or shuffling phase information of real EEG. We did not adopt the surrogate method because those methods construct surrogate for every experimental data from every lead and thus are very time-consuming. What is more, when we concern the phase information of signals, the meaning of conserving the same amplitude information or the same power spectrum, which is the core of aforementioned surrogate methods, is not that significant. In fact, in our previous study, we found that the threshold obtained via surrogate methods was almost the same as that obtained via filtering noise method. Therefore, we choose the filtering noise method in this manuscript. We believe that this method can be extended to other phase measures, and the most important requisite is that the filtered noise simulating series keep the same frequency band with the investigated signal.

**Simulation 1 .**

Cases of no phase locking.

*x*_1_(*t*) and *x*_2_(*t*) are, respectively, derived from *s*_1_ and *s*_2_, which are filtered from two independent normalized Gaussian white noises, that is,

(5) $$\begin{array}{c} x_{1}\left(t\right)=s_{1}\left(t\right), \end{array}$$

(6) $$\begin{array}{c} x_{2}\left(t\right)=s_{2}\left(t-\tau \right), \end{array}$$

in which *τ* represents time delay.  Figure 2 represents two instances of signal profiles and their corresponding phase series in simulation 1 when *τ* = 0 ms (Figure 2(a)), and *τ* = 100 ms (Figure 2(b)), respectively. As shown in Figure 2, although the oscillation frequencies are similar, maximums of linear correlation functions between *x*_1_ and *x*_2_, as well as between *φ*_1_ and *φ*_2_, are much less than 1, which means there is no obvious phase locking between *x*_1_ and *x*_2_, whatever does *τ* take. It is reasonable because *x*_1_ and *x*_2_ were derived from two independent sources.

**Simulation 2 .**

Cases of phase locking.

*x*_1_(*t*) and *x*_2_(*t*) are derived from the same *s*, which is filtered from Gaussian white noise, and *x*_2_(*t*) is delayed by *τ*, that is,

(7) $$\begin{array}{c} x_{1}\left(t\right)=s\left(t\right), \end{array}$$

(8) $$\begin{array}{c} x_{2}\left(t\right)=s\left(t-\tau \right). \end{array}$$

Figure 3 presents two instances of simulation 2 in case of *τ* = 0 ms (a) and *τ* = 100 ms (b). From both the waveform similarity and the linear correlation function maximum 1 or close to 1, we can see that there exits phase locking between *x*_1_ and *x*_2_. That makes sense because *x*_1_ and *x*_2_ are actually generated from the same source signal with a time delay.

The article "Classification for Memory Activities: Experiments and EEG Analysis Based on Networks Constructed via Phase-Locking Value" was published in 2022. Journal: Comput Math Methods Med.

In both simulation cases, *τ* varied from 0 to 500 ms, which is half of the series length, and PLVs between *x*_1_ and *x*_2_ were calculated for each *τ*. We independently repeated 100 times for each *τ* in both simulation cases, and the PLV statistics are listed in Table 1.

From Table 1, it can be seen that in simulation 1, when the two signals originate from independent sources, i.e., no phase locking, whatever the delay takes, the mean + SD of PLV is below 0.16, and there is no significant difference between different delays (two-sample *t*-test *p* > 0.05).

In simulation 2, when two signals originated from the same source signal, i.e., existing phase locking, PLV is greatly affected by the delay. To be specific, when *τ* = 0 ms, PLV exactly equals to 1, and it can be definitely differentiated from PLV obtained in simulation 1 with the same *τ*. As the delay increases, the PLV rapidly decreases, though, statistically significant difference between phase locking and non-phase locking keeps until *τ* = 25 ms (two-sample *t*-test *p* < 0.01). When the delay reaches 50 ms, PLV no longer takes significant difference between phase locking and non-phase locking (two-sample *t*-test *p* > 0.01). It shows that for signals with wide frequency band, PLV detects phase lock only when the delay is relatively short.

Then, we adopted the 95th percentage of PLV in simulation 1, i.e., 0.179, as the threshold for PLV binarization, and any PLV greater than this threshold will be considered phase locking. The underlying premise is that, with the support of simulation results, if PLV is greater than the threshold, there is only less-than-0.05 probabilities that there is no phase locking between the two signals of the same frequency band.

This method has a defect that it cannot identify phase locking with longer delay, e.g., delay longer than 25 ms in Gamma frequency band. Nevertheless, it sheds a light to phase-locking investigation between relatively wide-band signals.

## 4. Experiments

### 4.1. Experiment Design

The experiment was designed to investigate memory activities. Each subject sequentially underwent seven experimental steps, which took roughly an hour in total, as shown in Table 2.

In memory task experiment, we adopted the delayed match paradigm [28, 29], in which a target was first presented for three seconds, namely, memorization block, and then, after one-second gray screen with a cross at the center inducing still sight fixation, namely, retention block, a stimulus was presented for three seconds, i.e., match block. The subject was required to memorize the first target, retrieve it shortly to determine whether the stimulus was exactly the same as the memorized target, and click the corresponding option button, i.e., “yes” or “no,” as soon as the decision was made [30]. A sequence of a memorization block, a retention block, and a match block comprises a section, and 16 successive sections with 2 s break between two adjacent comprise a trial. Therefore, a trial lasts for 142 s.

The article "Classification for Memory Activities: Experiments and EEG Analysis Based on Networks Constructed via Phase-Locking Value" was published in 2022. Journal: Comput Math Methods Med.

The entire memory task experiment consists of four trials. In the same trial, the target and stimulus belong to the same category, e.g., colored digit series or colored character series, with fixed length. Furthermore, we modulate the memory load with series length. That is, in trials 1-3, in which both targets and stimulus were colored digit series, the series lengths were 1, , and 3, respectively. We took the assumption that the longer the series is, the heavier the memory load is. In addition, in trial 4, we used a colored English character as target as well as stimulus to investigate the difference between different target modalities, i.e., digit and character. The memory task experiment paradigm is illustrated in Figure 4.

As we can see, we cannot simply compare memory task experiment with rest condition to draw conclusion about memory, because subjects accept visual stimulus and make finger movement besides memorizing. Therefore, in order to focus on the memorizing activity as purely as possible, we also conducted the control experiment under the same paradigm as aforementioned. The only difference is that in the control experiment, the subject was not informed of the delayed match task but only asked to randomly click one of the two buttons, both with blank caption, every time the colored series following the cross showed up. We deliberately arranged the control experiment prior to memory task experiment, when subjects had no idea about the specific memory task, in order to get control states as pure as possible.

During experiments, both subjects' click moments and their choices (yes or no) were recorded by a background program, and then, each click was labeled “valid” or “nonvalid”; therein, a valid click was defined as the click happening after the stimulus showed up and before it faded away.

### 4.2. EEG Acquisition

The experiment was approved by the Ethics Committee of the Institutional Review Committee of the School of Electronic Science and Engineering of Nanjing University. All subjects were informed of the purpose as well as the content of the experiment and signed a consent. All experiments were carried out in the morning, between 09:00 and 12:00 am.

19 healthy subjects were enrolled in the experiment, including 18 male and 1 female with age of 23 ± 0.8 years old (mean ± SD). All of them were undergraduates or graduates; thus, they could understand the experiment instruction well. All subjects reported no drugs or alcohol taken in the last 24 hours. All subjects claimed right-handed and used their right hand to click the option button when necessary. Except that, other motions were discouraged.

The article "Classification for Memory Activities: Experiments and EEG Analysis Based on Networks Constructed via Phase-Locking Value" was published in 2022. Journal: Comput Math Methods Med.

During the experiment, the subject was seated in front of a 14′ monitor with a distance of approximate 40 cm, and both the target and the stimulus are presented at the center of the screen. All subjects reported clear sight with naked eyes or glasses on.

The Neuracle's 32-channel wireless EEG acquisition system (Neuracle Corp.) was used for 32-lead synchronized EEG acquisition. The electrode location conforms to the international 10-20 system, as shown in Figure 5. Sampling frequency was set 1000 Hz, and the impedance kept below 5 k*Ω* during the experiment.

### 4.3. EEG Preprocessing

The original signals were first 0.5-100 Hz band-pass filtered by “Basic FIR filter (new)” (Hamming window sinc FIR) in EEGLAB [31–33]. Then, the common mode interferences as well as artifacts were removed based on independent component analysis (ICA) [34]. In detail, we first adopted “run ICA” in EEGLAB [35], which is based on infomax algorithm. Then, for each decomposed component, we investigated vector angle *α* (method proposed by Li et al.) [36, 37] and kurtosis and removed those components with |cos(*α*)| ≥ 0.9 or kurtosis greater than 3. We also adopted amplitude threshold for spotting outliers based on interquartile range. Subsequently, 30-100 Hz Gamma rhythms were extracted through a fourth-order Butterworth filter with zeros ± 1. Following is segmentation, in which 1 s durations immediately prior to each valid clicking moment were extracted for following analysis. After preprocessing, we obtained 1 s slices of EEG which accompany the brain activity prior to finger clicking, and we expected them to reveal memorization activities. Preprocessing flow chart, as well as the EEG profile pre- and post-preprocessing, is presented in Figure 6.

Both in control and memory experiments, there were occasional missing clicks when the subject did not click any button during the required period. For these occasions, we not only left those missing clicks unsegmented but also discarded their counterpart in control or memory experiment of the same trial, considering the match demands in following analysis. And then, for every trial, we pooled all subjects together. The amount of valid EEG slices we finally retained is shown in Table 3.

The article "Classification for Memory Activities: Experiments and EEG Analysis Based on Networks Constructed via Phase-Locking Value" was published in 2022. Journal: Comput Math Methods Med.

## 5. Results and Discussion

### 5.1. Behavioral Data Analysis

We mainly investigated two behavioral indicators: memory accuracy (MA) and reaction time (RT), wherein the memory accuracy is defined as the percentage of correct choices made by the subject in each trial. And the reaction time is obtained through subtracting the stimulus moment from clicking moment.

We list the statistics of MA across 19 subjects in Table 4.

It can be seen that for all trials, MAs in memorization experiments are significantly higher than those in control, which indicates that subjects indeed focused on memorization tasks as required.

Then, we list the statistics of RT across 19 subjects in Table 5. Note that visual targets in the control and memory experiment were exactly the same; subject- and section-matched RT variations from control to memory task, as well as *p* values of *t*-tests for subject- and section-matched RT variations, are listed in the last two columns of Table 5.

From Table 5, it can be seen that in trials 2 and 3, it took significantly shorter time for subjects to act under control conditions than under memorization ones, with *t*-test *p* values being less than 0.01. It implies less mental effort of subjects under control than memorization, as the experiment was designed. Nevertheless, as for trial 1 and trial 4, RTs under control were not significantly shorter. A potential reason is the start or switch effect; that is, trial 1 was the very beginning of all behavioral experiments, when subjects were not yet skilled enough with what they were expected to do; thus, it took time to get familiar, and in trial 4, we converted the visual target from digits to letters, which also demanded the subject's adaption.

We also conducted two-sample *t*-test of RTs between every two trials and listed *p* values in Table 6.

It can be seen that under control, except for trial 1 vs. 2 and 3, there is no significant difference in RT (*p* > 0.01), and even the significant differences between trial 1 vs. 2 and trial 1 vs. 3 might result mainly from the start effect aforementioned. As for memorization condition, there is no significant difference in RT between different trials observed (*p* > 0.01). It implies that, although the memory load or target form varied, RT was not affected significantly, at least under temporary precision of this research. In fact, under current experimental paradigm, subjects' activities of recollecting, decision, and finger movement cannot be clearly separated in temporal axis that is a potential reason for significant difference absence in Table 6.

The article "Classification for Memory Activities: Experiments and EEG Analysis Based on Networks Constructed via Phase-Locking Value" was published in 2022. Journal: Comput Math Methods Med.

### 5.2. EEG Classification Results

For each temporary slice, treating each channel (electrode or lead) in 32 channels as a separate node, we calculated the PLV between every two channels. Then, based on the threshold setup in simulation, we conducted the binarization, resulting in 0 representing no phase locking and 1 representing phase locking. After that, brain functional networks were constructed and the node degree, clustering coefficient, and betweenness centrality for each lead were extracted; thus, we obtained 96 features for each EEG slice. Subsequently, they were used as a 96-dimention inputting vector and inputted into the SVM for classification. We took four classification tasks:

Classification task 1

After pooling all trials together, we tried to distinguish memorization from control, regardless of different memory loads or target forms. As shown in Table 3, sample size in this task is 2292, with one-half memorization and one-half control.

Classification task 2

Focusing on trial 3, in which the memory load was designed heaviest and differences between control and memorization experiment were expected greatest, we tried two-category classification, i.e., memorization or control. As shown in Table 3, sample size in this task is 570, including 285 for each category.

Classification task 3

For memorization experiments in trials 1 and 4, we tried to discern difference between different target forms, which was still a two-category classification, i.e., digit target or character one. As shown from Table 3, sample size in this task is 574, including 286 digit-target cases and 288 letter-target cases, respectively.

Classification task 4

For memorization experiments in trials 1, 2, and 3, in which the same kind of target forms was represented, i.e., colored digit series, we tried three-category classification to distinguish different memory loads. As drawn from Table 3, sample size in this task is 858, specifically 286, 287, and 285 for light, medium, and heavy memory load, respectively.

For all four classification tasks, we first pooled all slices from all subjects together, randomly shuffled them, and then randomly split them into training set and testing set according to ratio 7 : 3. Subsequently, we trained our model on training set with tenfold cross-validation. Grid-searching was adopted in tenfold cross-validation in training to help determine penalty factor *C* and kernel function parameter *γ*. It turned out that best parameter set varied from task to task. Then, we applied the obtained best models to corresponding test sets. Performance evaluations [38, 39] for tasks 1, 2, and 3 are listed in Table 7, and those for task 4 are listed in Table 8.

The article "Classification for Memory Activities: Experiments and EEG Analysis Based on Networks Constructed via Phase-Locking Value" was published in 2022. Journal: Comput Math Methods Med.

From Tables 7 and 8, it can be seen that our models achieve satisfactory performance in general. Specifically, the classification accuracy in task 1 is the lowest while that in task 3 is the highest. Considering that in task 1, we included all four trials with no regard of memory loads or target forms, it is quite reasonable that the complex data-comprising would complicate the classification. On the contrary, as for task 2 as well as 3, when datasets comprise fewer variable factors, the model works better.

It is also inspiring that the model has a decent performance when distinguishing different memory loads. In BCI or neural feedback, quantification of brain effort is really important, although it is difficult. Our model provides a promising solution to brain effort quantification.

### 5.3. Most Important Characteristic Visualization and Interpretation

We then investigated the permutation importance [41] in SVM of 96 characteristics and found that their distribution is significantly different from a uniform or normalization distribution (*p* of KS tests far less than 0.01), and certain characteristics that ranked within top 10 are far away from the rest. It implies that these characteristics are much more crucial than the other in classification. It is interesting that almost all most important characteristics are node degrees. We infer that the small-world-network traits, represented by local clustering coefficient and betweenness centrality, do not dominate the difference between memorization and control, neither among different memory loads or target forms, considering that all features input into SVM have been normalized. In order to get a visualization, in Figure 7, we presented the topographic maps of differences of these most important characteristics (a) between control and memorization under memory load 3, (b) between memorizing English character and memorizing digit, and (c) between memory load 1 and load 3, respectively, with exaggerating the circle size of the node and color representing the difference intensity, in more detail.

For data in task 2, we calculated variations from control to memory with the heaviest memory load for each matched section, i.e., subtracting values under control from values under memorization of exactly the same visual presentation. Then, we took the arrhythmic means across the dataset and mapped them to colors in the circle representing the lead/node location, resulting in Figure 7(a).

For data in task 3, we calculated difference of the most important node degrees between trial 1 (digit target) and trial 4 (English character target), i.e., subtracting group-average under trial 1 from that under trial 4. Then, we mapped them to colors in the circle representing the lead/node location, resulting in Figure 7(b).

The article "Classification for Memory Activities: Experiments and EEG Analysis Based on Networks Constructed via Phase-Locking Value" was published in 2022. Journal: Comput Math Methods Med.

For data in task 4, we also present difference between different memory loads in Figure 7(c); that is, we subtract group average of the most important node degree under memory load 1 from that under load 3; then, we mapped them to colors in the corresponding circle.

We did not visualize task 1 because it is hard to interpret considering that in task 1, we mixed together different variables, i.e., memory targets as well as memory loads.

From Figure 7, we find some interesting and meaningful phenomenon.

Under the heaviest memory load with digit target form, node degrees of Cz and F8 are most obviously enhanced when memorization compared with the control stage, and node degrees of FP1 and F7 are most obviously weakened. Considering that Cz has been widely applied to attention feedback/training to track attention level in real time [42], it is reasonable that Cz functions more actively in memory than in control, resulting in node degree of Cz increasing. In addition, according to Okamoto and colleague's work on correlation between the international 10–20 system and Brodmann Area (BA) [43]; FP1, F7, and F8 correspond to BA9 and BA10, which are believed responsible for working memory, attention, and task management and planning [44, 45]. Therefore, topography (Figure 7(a)) shows consistency with the underlying brain function during memory task in certain degrees. As to the opposite variation between F7 and F8, we speculate that it might result from the ipsilateral increment and the contralateral decrement, since all subjects reported right-handed.

When comparing character memorization with digit memorization (Figure 7(b)), the node degree enhancement in T7 is most impressive. It is interesting that T7 corresponds most to BA 21 [43], which is in charge of semantic memory processing and language processing besides visual perception [44, 45]. Therefore, it partly supports that the brain does process character and digit in different ways and treat character as language even there is only one character.

As to variation from the lightest memory load to the heaviest with the same target form of digit (Figure 7(c)), node degree increments of T8, P8, CP6, and C4 combined with decrement of F7 are most obvious. Corresponding to T8, P8, CP6, and C4 are BA 19-22, as well as BA39 [43], in which BA19-22 are related with visual perception, processing, and memory [44, 45]. It is worth noting that BA39, which only resides in the right hemisphere, is believed responsible for number processing. We infer that the longer the digit series length is, the more active the BA39 function is, which is represented by the higher node degree.

The article "Classification for Memory Activities: Experiments and EEG Analysis Based on Networks Constructed via Phase-Locking Value" was published in 2022. Journal: Comput Math Methods Med.

Nevertheless, since there are only 19 subjects and the memory task design needs further improvement, e.g., difference between adjacent memory loads should be designed greater, more experiments are required for further uncovering the neural mechanism of memory.

## 6. Conclusion

In this work, we designed and conducted series of experiments concerning memory and collected behavioral data as well as 32-lead EEG signals simultaneously. Combined with behavioral data analysis, we segmented EEG signals into slices; then, we calculated Gamma rhythm PLV between every two leads, conducted binarization, constructed brain function network, and extracted three network characteristics of node degree, local clustering coefficient, and betweenness centrality. Subsequently, we inputted these network characteristics of all leads into SVMs for classification and obtained decent performances. Based on the result, we believe that network characteristics based on binarized PLV have the ability to distinguish the presence or absence of memory, as well as the intensity of the mental workload at the moment of memory. Finally, we tried visualizing the difference of those characteristics ranking top in SVM permutation importance for three representative contrasts and obtained intuitive topographic maps. The obtained topographic maps provide information that is consistent with neurophysiology in certain degrees.

It is worth noting that PLV was not suitable for wide-band signals, which is the case for Gamma rhythm. In order to resolve this problem, we proposed using filtered noise of the same frequency band with Gamma rhythm as simulating series to obtain the binarization threshold. This method can sensitively detect phase locking with temporary delay no longer than 25 ms. However, it is also the limitation of the method.

## Figures and Tables

**Figure 1:** The overall flow chart of the method.

**Figure 2:** Two instances of signal profiles and corresponding phase series in simulation 1.

**Figure 3:** Two instances of signal profiles and corresponding phase series in simulation 2.

**Figure 4:** Illustration of the memory task experiment paradigm. Every experiment consists 4 trials, each trial includes 16 sections, and each section includes 3 blocks of 3 s memorization block, 1 s retention block, and 3 s match block sequentially. In trials 1-3, both the target and the stimulus are colored digit series, with lengths 1, 2, and 3, respectively, corresponding to ascending memory loads. In trial 4, both targets and stimulus are colored English characters, representing a different target modality.

The article "Classification for Memory Activities: Experiments and EEG Analysis Based on Networks Constructed via Phase-Locking Value" was published in 2022. Journal: Comput Math Methods Med.

**Figure 5:** Channel locations.

**Figure 6:** Preprocessing flow chart and EEG profiles before and after preprocessing.

**Figure 7:** Three representative topographic maps of differences between two states for node degrees ranking the most important in permutation importance. (a) Difference between control and memorization under memory load 3. (b) Difference between memorizing English character and memorizing digit. (c) Difference between memorization under memory load 3 and under load 1. Circle sizes of these most important nodes are exaggerated for clear sight. Warm color represents increment, while cool color represents decrement.

**Table 1:** PLV statistics of 100 independent experiments in simulation.

*τ* (ms)	PLV (mean ± SD) Simulation 1: no phase lock	PLV (mean ± SD) Simulation 2: phase lock	*p* value of two-sample *t*-test between simulation 1 and 2
0	0.094 ± 0.049	1.000 ± 0.000	1.985 × 10^−127^
5	0.094 ± 0.043	0.729 ± 0.026	6.459 × 10^−145^
10	0.095 ± 0.047	0.338 ± 0.060	3.081 × 10^−59^
25	0.089 ± 0.048	0.155 ± 0.066	0.004
50	0.096 ± 0.045	0.098 ± 0.055	0.062
100	0.096 ± 0.049	0.101 ± 0.051	0.367
200	0.098 ± 0.049	0.096 ± 0.051	0.843
500	0.097 ± 0.054	0.089 ± 0.051	0.740

**Table 2:** Experimental process.

Step	Operator activities	Subject activities	Rough duration (min)
(1) Information	Inform subjects of the general aim and rough content of the experiment	Sign the consent and fill the questionnaire.	3
(2) Setup	EEG cap placement with gel infusion, acquisition setup, and time calibration	Be seated.	20
(3) Rest baseline	EEG monitoring and acquisition	Be seated in quiet and relaxed manner, with eyes open.	2
(4) Control instruction	Inform subjects of what they are expected to do in the immediately following step	Understand the instruction and communicate, if necessary, to avoid ambiguousness.	2
(5) Control experiment	EEG monitoring and acquisition	Act as instructed.	15
(6) Memory task instruction	Inform subjects of what they are expected to do in the immediately following step	Understand the instruction and communicate, if necessary, to avoid ambiguousness.	2
7.Memory task experiment	EEG monitoring and acquisition	Act as instructed.	15

**Table 3:** The amount of valid EEG slices in each trial.

	Control	Memory experiment	Row total
Trial 1	286	286	572
Trial 2	287	287	574
Trial 3	285	285	570
Trial 4	288	288	576
Column total	1146	1146	2292

**Table 4:** Statistics of MA across 19 subjects.

	MA under control condition (mean ± SD)	MA under memorization (mean ± SD)	Subject-matched MA variation (memory-control) (mean ± SD)	*p* of *t*-test for subject-matched MA variations
Trial 1	0.536 ± 0.138	0.984 ± 0.027	0.448 ± 0.135	2.74 × 10^−7^
Trial 2	0.552 ± 0.137	0.932 ± 0.069	0.380 ± 0.126	7.44 × 10^−7^
Trial 3	0.573 ± 0.127	0.984 ± 0.027	0.411 ± 0.143	1.19 × 10^−6^
Trial 4	0.563 ± 0.165	1.000 ± 0.000	0.438 ± 0.165	2.68 × 10^−6^

The article "Classification for Memory Activities: Experiments and EEG Analysis Based on Networks Constructed via Phase-Locking Value" was published in 2022. Journal: Comput Math Methods Med.

**Table 5:** Statistics of RT across 19 subjects.

	RT under control condition (mean ± SD) (ms)	RT under memorization condition (mean ± SD) (ms)	Subject- and section-matched RT variation (mean ± SD) (ms)	*p* of one-sample *t*-test for subject- and section-matched RT variations
Trial 1	687.5 ± 689.0	692.7 ± 695.5	5.200 ± 904.3	0.937
Trial 2	484.4 ± 661.0	692.7 ± 563.0	208.3 ± 720.5	9.180 × 10^−5^
Trial 3	411.5 ± 663.3	828.1 ± 893.6	416.6 ± 868.0	3.280 × 10^−10^
Trial 4	531.3 ± 816.0	661.4 ± 641.4	130.2 ± 871.3	0.040

**Table 6:** *p* values of two-sample *t*-test of RTs between every two trials.

	Control	Memorization
Trial 1 vs. 2	0.003	1.000
Trial 1 vs. 3	8.000 × 10^−5^	0.099
Trial 1 vs. 4	0.044	0.648
Trial 2 vs. 3	0.283	0.077
Trial 2 vs. 4	0.538	0.613
Trial 3 vs. 4	0.116	0.037

**Table 7:** Performance evaluations for two-category classification of tasks 1, 2, and 3.

Task	*c*	*γ*	Accuracy in test set	Precision in test set	Recall in test set	AUC_ROC in test set
1	5	1	0.782	0.788	0.782	0.857
2	50	1	0.830	0.798	0.864	0.910
3	5	0.5	0.895	0.870	0.904	0.946

**Table 8:** Performance evaluations for three-category classification of task 4.

Task	*C*	*γ*	Indicator type	Accuracy in test set	Precision in test set	Recall in test set	AUC_ROC in test set
4	50	0.5	class0	0.808	0.828	0.750	0.903
			class1		0.772	0.830	0.926
			class2		0.825	0.855	0.945
			Micro^∗^		0.808	0.808	0.923
			Macro^∗∗^		0.808	0.812	0.925

^∗^Micro evaluators are globally calculated by counting the total true positives, false negatives, and false positives. ^∗∗^Macro evaluators are directly obtained by unweighted averaging metrics from all classes [40].

## Data Availability

The labeled dataset used to support the findings of this study is available from the corresponding author upon request.
